The article "Phillygenin Protects the Intestinal Barrier from Dysfunction via let-7b Signaling Pathway and Regulation of Intestinal Microbiota" was retracted in 2023. Reasons: signs of a paper mill; suspected computer-generated content; unreliable results or conclusions; lack of ethics approval or compliance.

# Phillygenin Protects the Intestinal Barrier from Dysfunction via let-7b Signaling Pathway and Regulation of Intestinal Microbiota

**DOI:** 10.1155/2022/4769709

**Published:** 2022-03-16

**Authors:** Huiping Feng, Ling He, Zihua Wang, Bin Pi, Zhihua Liu

**Affiliations:** ^1^Department of Clinical Nutrition, The Fifth Affiliated Hospital of Guangzhou Medical University, Guangzhou, Guangdong 510799, China; ^2^Department of AnoRectal Surgery, The Fifth Affiliated Hospital of Guangzhou Medical University, Guangzhou, Guangdong 510799, China; ^3^Department of Emergency, The Fifth Affiliated Hospital of Guangzhou Medical University, Guangzhou, Guangdong 510799, China

## Abstract

The study investigates the positive effects of phillygenin on intestinal tight junction via the let-7b signaling pathway and the regulation of intestinal microbiota. The expression levels of tight junction proteins are determined through PCR and Western blot. DSS-induced mice colitis is used to verify the protective effects of phillygenin on intestinal barrier and tight junction. Fecal microbiota transplantation is used to verify the role intestinal microbiota. let-7b is detected in the colon tissues of patients with acute stercoral obstruction. Phillygenin could promote the expression of occludin, which might be inhibited by let-7b inhibitor. DSS-induced mice colitis showed that phillygenin could lower the colonic permeability and maintain the tight junction-associated proteins. The effects of phillygenin could be deprived by anti-let-7b and rescued by FMT of normal intestinal microbiota. Clinical samples verified a lower level of let-7b in stercoral obstruction patients. Phillygenin could protect the intestinal barrier from dysfunction via the signaling pathway of let-7b by regulating intestinal microbiota.

## 1. Introduction

Recently, various studies focused on the intestinal mucosa barrier dysfunction (IMBD) and dysbiosis of intestinal microbiota [1, 2]. However, effective drugs and the treatment methods still need to be further investigated [3]. It is reported that phillygenin is an important active ingredient of lignans with a fingerprint component in Forsythiae Fructus [4]. Furthermore, it is reported as a wide-used protector with various functions, such as antiviral, antioxidant, anti-inflammatory, anticancer, and antifibrosis effects [4–8]. MicroRNAs (miRs) are mainly negative regulators of their target genes through binding to 3'untranslated regions (3'UTRs) [9–12]. miRs could regulate the expression of target genes, through inhibiting the mRNA translation, or by causing mRNA degradation. miRNAs are reported to be associated with intestinal diseases as well. Studies about miRs, intestinal barrier function, and intestinal microbiota are popular. McKenna et al. found that intestinal barrier dysfunction could be induced in the Dicer1-conditional knockout mice, with lymphocytes and neutrophils infiltrating in colon. Liu et al. investigated the role of miR-155 on intestinal barrier in the dextran sulfate sodium (DSS)-induced mice colitis, indicating that miR-155 inhibitor could relieve weight loss and intestinal damage. miR-21 could protect the intestinal barrier function and higher the expression of tight junction-associated proteins via the Rho-ROCK signaling pathway of ROCK-1 [2].

In our previous study, let-7b is identified to protect intestinal barrier function, and negative regulation of p38 MAPK signaling is involved in the protective process. One study about phillygenin found that it could improve inflammation and fibrosis of the liver caused by CCl_4_, through promoting ZO-1, occludin, and claudin-1. However, the effects and molecular mechanism of phillygenin during the therapeutic process of intestinal barrier dysfunction have not been reported. In this study, we aim to investigate the molecular mechanisms of phillygenin about the protective effects of the intestinal epithelial barrier through the pathway of let-7b.

## 2. Our Proposed Method

### 2.1. Cell Culture

Caco-2 cells are grown in Dulbecco's modified Eagle medium (DMEM, Gibco, Life Technologies) supplemented with 10% FBS, 100 U/ml penicillin, and 100 ug/ml streptomycin at 37°C in a humidified atmosphere containing 5% CO_2_. Cell passage is performed using 0.05% trypsin and 0.5 mm EDTA (Gibco, USA) as previously described. Phillygenin is purchased from the Chengdu Must Biotechnology Co., Ltd. Lentivirus vectors or inhibitors are constructed by Shanghai Minzai Co., Ltd. The Caco-2 cells are transfected with Lipofectamine 2000 (Invitrogen, USA).

### 2.2. DSS-Induced Mice Colitis

As described, mice colitis is induced by adding 3.0% DSS (36–50 kDa; MP Biomedicals) in their drinking water for seven days. Animals are sacrificed after collecting blood from their eyeballs, and colons are prepared for histological analysis. Mice in the phillygenin groups are given 20 mg/kg phillygenin via oral gavage once a day, respectively. As for the intraperitoneal injection, 10 *μ*g of let-7b inhibitor in 100 *μ*l sterile saline is administered. For fecal microbiota transplantation (FMT), fecal microbiota of WT mice is transplanted to mice with colitis, especially for mice treated with anti-let-7b to investigate the therapeutic effects of phillygenin and let-7b. Stools from donor mice are collected under a laminar flow hood in sterile conditions and 100 mg stool is suspended in 3 ml of sterile saline. The solution is vigorously mixed and centrifuged at 2000 g for 3 min. The deposit is resuspended in 3 ml of sterile saline and used as the transplant material. Fresh transplant material is prepared on the same day of transplantation within 10 min before oral gavage (300 mg/kgBW). Recipient mice are inoculated every other day for 2 weeks before being killed for subsequent analysis.

### 2.3. Permeability Assay

To evaluate the permeability of Caco-2 cells and DSS-induced mice colitis, measurement of transepithelial electrical resistance (TER) and dextran permeability is determined as reported previously. The fractional excretion for sucralose is determined to evaluate the colonic permeability, while the ratio of fractional excretion for lactulose/mannitol is used to detect the small intestinal permeability. Using chamber assay is also an indicator to evaluate the intestinal permeability, using the isolated mice colons as reported.

### 2.4. Quantitative Real-Time Polymerase Chain Reaction (qRT-PCR) Analysis

Total RNA is extracted from cells or tissue samples using TRIzol lysis buffer (Ambion, USA) according to the manufacturer's instructions. The microRNA isolation of cell or tissue or serum samples is performed with the miRNeasy Mini Kit (Qiagen, Germany) according to the manufacturer's instructions. First strand synthesis of cDNA is performed with the reverse transcription kit (Invitrogen, USA). A qRT-PCR for mRNA is performed using SYBR Master Mix (Invitrogen, USA) and using a 7500 Real-Time PCR system.

Western blotting is performed by a wet electroblotter (Bio-Rad) for 120 min at 100 V as previous reported [1, 2]. The membrane is detected by the enhanced chemiluminescence method (ECL kit; Pierce, Illinois) according to the manufacturer's instructions. Serum and tissue samples of acute stercoral obstruction patients are used to evaluate the expression level of miRNA. Fresh colon and serum are collected from the stercoral obstruction patients. Colon and the paired adjacent normal colon tissues are used to determine the expression levels of miRNA and related inflammatory factors. Tissues are collected from patients in The Fifth Affiliated Hospital of Guangzhou Medical University, which is approved by the Scientific and Ethical Committee of The Fifth Affiliated Hospital of Guangzhou Medical University in accordance with the approved human subject guidelines. Statistical data are analyzed by GraphPad Prism 5 software (San Diego, CA) and expressed as mean ± SEM. Statistical analysis is performed using Student's *t*-test. *P* value <0.05 is defined as significant.

## 3. Clinical Experimental Results

### 3.1. Phillygenin Could Alleviate Occludin Decrease Induced by let-7b Inhibitor in Caco-2 Cells

To determine the effects of phillygenin, the Caco-2 cell line is transfected with let-7b inhibitor. Results indicated that let-7b expression is significantly decreased, compared with the control (*P* < 0.05), as shown in Figure 1(a). Although LPS might inhibit the expression of TJ-associated protein occludin in Caco-2 cells, occludin is promoted after the pretreatment of phillygenin, while let-7b inhibitor could deprive the protective effects of phillygenin (*P* < 0.05), as shown in Figure 1(b). Western blot analysis showed same results, as shown in Figure 1(c).

### 3.2. Phillygenin Could Lower the Expression of p38 MAPK via let-7b

To further investigate the molecular mechanism of phillygenin and its molecular mechanism, we investigated the expression p38 MAPK by qRT-PCR with the transfection of let-7b inhibitor or precursor. Phillygenin could inhibit the expression of P38 MAPK in Caco-2 cells, compared with the LPS group; however, let-7b inhibitor could disrupt the decrease of P38 MAPK after transfection into the Caco-2 cells (*P* < 0.05), as shown in Figure 2(a). In contrast, after let-7b precursor is transfected into Caco-2 cells, p38 MAPK signaling also fell significantly, with or without the pretreatment of phillygenin (*P* < 0.05), as shown in Figure 2(b).

### 3.3. Phillygenin Could Alleviate the DSS-Induced Mice Colitis via let-7b and Intestinal Microbiota

Intestinal permeability is investigated to verify the protective effects of phillygenin on intestinal barrier. TER level significantly decreased after treatment of phillygenin in Caco-2 cells (*P* < 0.05), as shown in Figure 3(a). While the relative intensity rose, however, transfection of let-7b inhibitor could inhibit the effects of phillygenin (*P* < 0.05), as shown in Figure 3(b). Using chamber assay indicated that phillygenin could lower the intestinal permeability of mice; however, injection of anti-let-7b could deprive the effects of phillygenin, and FMT from the control group could inhibit the effects of anti-let-7b (*P* < 0.05), as shown in Figures 3(c) and 3(d). The lactulose/mannitol rate and sucralose excretion increased in the DSS-induced mice colitis, which is relieved by phillygenin and rescued by FMT after injection of anti-let-7b as well (*P* < 0.05), as shown in Figures 3(e) and 3(f).

The average body weight of DSS-induced mice is lower than control, which could be relieved by giving phillygenin in drinking water; however, intraperitoneal injection of anti-let-7b could lower the bodyweight of mice and FMT would also retain the bodyweight (*P* < 0.05), as shown in Figure 4(a). The qRT-PCR assays revealed that serum IL-6, TNF-*α*, and zonulin levels increased in the DSS-induced mice colitis group, compared to the WT group significantly, which are relieved by drinking phillygenin. However, the serum factors reincreased by intraperitoneal injection of anti-let-7b and inhibited by FMT from WT mice (*P* < 0.05), as shown in Figures 4(b)–4(d). Determination of occluding and ZO-1 in colon tissues also indicated a significant decrease of expression levels of the two TJ proteins in the DSS-induced mice colitis group, while the effects could be relieved by giving the drugs of phillygenin to mice, and the inhibiting effects of anti-let-7b would also be prevented by FMT from WT mice (*P* < 0.05), as shown in Figures 4(e) and 4(f). The expression level of let-7b is also evaluated, which indicated that phillygenin could enhance the expression of let-7b in the DSS-induced mice colitis model; whereas, FMT did not impact the expression of let-7b (*P* < 0.05), as shown in Figure 4(g).

### 3.4. Low Levels of let-7b Are Detected in Clinical Samples of Acute Stercoral Patients

let-7b in colon tissues of stercoral obstruction patients significantly decreased than control (*P* < 0.05), as shown in Figure 5(a). Occludin and Zo-1 expression levels from fresh tissues also decreased significantly, compared with control (*P* < 0.05), as shown in Figures 5(b) and 5(c). Meanwhile, serum inflammatory factors, such as zonulin, IL-6, and TNF-*α*, increased through the determination of the ELISA kit (RayBiotech, USA) in patients with intestinal barrier dysfunction of stercoral obstruction (*P* < 0.05), as shown in Figures 5(d)– 5(f).

## 4. Experimental Result Analysis

In our study, we investigated phillygenin on intestinal barrier dysfunction via the let-7b/p38 MAPK signaling pathway. Results indicated that phillygenin could activate the let-7b/P38 MAPK pathway in Caco-2 cells and show its therapeutic effects on intestinal mucosal barrier dysfunction. Determination of mice showed the positive effects of phillygenin on intestinal barrier and tight junction-associated proteins, such as occludin and ZO-1, via the let-7b/p38 MAPK signaling pathway. Clinical samples verified the decline of let-7b in patients with intestinal barrier dysfunction of acute stercoral obstruction. Phillygenin could higher the occluding expression after the pretreatment of LPS in Caco-2 cells; while transfection, the let-7b inhibitor could significantly inhibit the effects of phillygenin. It is reported that let-7b might play a positive role on intestinal barrier function by targeting p38 MAPK. We hypothesized that phillygenin could protect intestinal barrier from dysfunction through the let-7b/MAPK signaling pathway. Our study indicated that let-7b inhibitor could promote p38 MAPK expression, compared with the single phillygenin group. In contrast, the expression level of P38 MAPK is inhibited by let-7b precursor in Caco-2 cells. Moreover, we further verified the role of phillygenin and let-7b in the mice model and clinical samples of stercoral obstruction patients. Our study indicated that let-7b might be one of the important molecular mechanisms of phillygenin during the protection process of intestinal barrier dysfunction induced by DSS because the let-7b inhibitor could alleviate the effects of phillygenin about the decrease of the intestinal permeability in vitro and in vivo. Furthermore, phillygenin could also inhibit the inflammatory factors and maintain occluding and Zo-1, as well as promote the expression level of let-7b. In order to further verify the effects of intestinal microbiota, we further gave the pretreatment of intraperitoneal injection of anti-let-7b and found the protective effects of phillygenin are inhibited by anti-let-7b. However, when the mice are transplanted with the normal stool, the protective effects of phillygenin are rescued by the FMT method. Meanwhile, the expression level of let-7b is not impacted by FMT. Therefore, the results indicated that intestinal microbiota exerted important effects during protection of IMBD. Clinical samples are also detected, and results indicated that inflammatory factors, such as IL-6 and TNF-*α*, are increased significantly in the colonic tissues of acute stercoral obstruction patients, while let-7b, occludin, and ZO-1 are all decreased. One study showed that Crohn's disease-associated adherent invasive *Escherichia coli* could elicit and exacerbate colitis in IL-10 KO mice, by injury the intestinal barrier and lower the tight junction associated proteins. Proinflammatory cytokines of T84 cells, such as IL-6 and TNF-*α*, maybe caused by TLR4 overexpression and let-7b inhibition. let-7b significantly ameliorated the mice colitis and reduced the secretion of inflammatory cytokines through TLR4. Another study showed that phillygenin could improve inflammation and fibrosis caused by CCl_4_ [4]. Furthermore, it restored the intestinal barrier by promoting ZO-1, occludin, and claudin-1. Phillygenin enriches the relative abundance of *Lactobacillus* and regulated the intestinal microbiota, which are reported to effectively alleviate the intestinal barrier injury [4]. Recent study also found that phillygenin also inhibited LPS-induced inflammation through TLR4/MyD88 signaling and suppress the adaptive immune response and inflammatory activities. However, the study about the relationship between phillygenin and IMBD has not been reported. In our study, we mainly investigated the protective effects of phillygenin from intestinal barrier dysfunction via the let-7b/P38MAPK signaling pathway through the regulation intestinal microbiota. One limitation of our study may be that we have no direct evidence to verify the therapeutic effects of phillygenin on the intestinal barrier function and its impaction on let-7b expression. Whether there are some middle molecular mechanisms and pathways or other key moleculars should also be studied as well. Further studies or proper clinical trials might be needed to verify this hypothesis.

## 5. Conclusion

In conclusion, phillygenin could protect intestinal barrier from dysfunction via let-7b signaling by regulation of intestinal microbiota. The molecular mechanism may be that phillygenin might inhibit the let-7b/P38 MAPK pathway.

The study investigates the positive effects of phillygenin on intestinal tight junction via the let-7b signaling pathway and the regulation of intestinal microbiota. The expression levels of tight junction proteins are determined through PCR and Western blot. DSS-induced mice colitis is used to verify the protective effects of phillygenin on intestinal barrier and tight junction. Fecal microbiota transplantation is used to verify the role intestinal microbiota. let-7b is detected in the colon tissues of patients with acute stercoral obstruction. Phillygenin could promote the expression of occludin, which might be inhibited by let-7b inhibitor. DSS-induced mice colitis showed that phillygenin could lower the colonic permeability and maintain the tight junction-associated proteins. The effects of phillygenin could be deprived by anti-let-7b and rescued by FMT of normal intestinal microbiota. Clinical samples verified a lower level of let-7b in stercoral obstruction patients. Phillygenin could protect the intestinal barrier from dysfunction via the signaling pathway of let-7b by regulating intestinal microbiota.

## Figures and Tables

**Figure 1:** Phillygenin could alleviate decrease of occludin expression induced by let-7b inhibitor. (a) Analysis of the relative expression level of let-7b determined by qRT-PCR in Caco-2 cells transfected with let-7b inhibitor and control. (b) LPS could lower the expression of occludin in Caco-2 cells. However, after the pretreatment of phillygenin, expression of occludin is increased, while let-7b inhibitor deprived the effects of phillygenin. (c) Western blot analysis showed same effects of phillygenin and let-7b as qRT-PCR. ^*∗*^ vs. the LPS group, *P* < 0.05, ^*∗*^ vs. ^#^, *P* < 0.05.

**Figure 2:** Phillygenin downregulated the p38 MAPK signaling and inhibited by let-7b inhibitor. (a) LPS could higher the expression of p38 MAPK in Caco-2 cells significantly, and phillygenin could inhibit the effects of LPS; however, after let-inhibitor is transfected, P38 MAPK expression rose. (b) Analysis of the relative expression level of P38 MAPK at mRNA level inlet-7b transfected Caco-2 cells and control with or without the pretreatment of phillygenin. ^*∗*^ vs. the LPS group, *P* < 0.05, ^*∗*^vs ^#^, *P* < 0.05.

**Figure 3:** Phillygenin could lower intestinal permeability through the inhibition of let-7b and ROCK-1 pathways. (a) Transepithelial electrical resistance is lowered after the pretreatment of phillygenin in Caco-2 cells, which could be relieved by the transfection of let-7b inhibitor. (b) The relative intensity is enhanced after the pretreatment of phillygenin, which could be relieved by transfection of let-7b inhibitor. (c) Mannitol flux is increased in the DSS-induced mice colitis group, compared with the control wild-type group, which could be relieved by phillygenin. The effects of phillygenin could be deprived by anti-let-7b and rescued by FMT of normal intestinal microbiota. (d) The resistance is decreased in the DSS-induced mice colitis group, compared with the control wild-type group, which could be relieved by phillygenin. The effects of phillygenin could be deprived by anti-let-7b and rescued by FMT of normal intestinal microbiota. (e) The lactulose/mannitol rate is higher in the DSS-induced mice colitis, compared with the control WT group at 8 and 12 week mice, which could be relieved by phillygenin. The effects of phillygenin could be deprived by anti-let-7b and rescued by FMT of normal intestinal microbiota. (f) The sucralose excretion is higher in the DSS-induced mice colitis group, compared with the control WT group at 8 and 12 week mice in vivo, which could be relieved by phillygenin. The effects of phillygenin could be deprived by anti-let-7b and rescued by FMT of normal intestinal microbiota. ^*∗*^ vs. control. ^*∗*^ vs. ^#^, ^#^ vs. ^*∗∗*^, ^*∗∗*^ vs. ^##^, *P* < 0.05. Three independent experiments are performed for the cell test, and fifteen are performed for mice.

**Figure 4:** Phillygenin could relieve the destruction of tight junction. (a) Bodyweight of DSS-induced mice is lower; while after the pretreatment of phillygenin, the bodyweight became higher compared with the DSS group. The effects of phillygenin could be deprived by anti-let-7b and rescued by FMT of normal intestinal microbiota. (b)–(d) Serum levels of zonulin, IL-6, and TNF-*α* levels are higher in the DSS-induced mice colitis group, compared with the WT group, which could be relieved by anti-ROCK-1. The effects of phillygenin could be deprived by anti-let-7b and rescued by FMT of normal intestinal microbiota. (e)-(f) Occludin and ZO-1 of colon tissues decreased in the DSS-induced mice colitis group, while the effects could be relieved by giving the drugs of phillygenin to mice. The effects of phillygenin could be deprived by anti-let-7b and rescued by FMT of normal intestinal microbiota. (g) Phillygenin could enhance the expression of let-7b in the DSS-induced mice colitis model. FMT did not impact the expression level of let-7b. ^*∗*^ vs. control, ^*∗*^ vs. ^#^, ^#^ vs. ^*∗∗*^, ^*∗∗*^ vs. ^##^, *P* < 0.05. Three independent experiments are performed for the cell test, and fifteen are performed for mice.

**Figure 5:** Detection of the clinical samples of acute stercoral obstruction patients to evaluate the levels of miR-155, occluding, and Zo-1 in colon tissues and zonulin, IL-6, and TNF-*α* in serum. (a) The expression levels of let-7b decreased in the stercoral obstruction group, compared with paired obstruction-adjacent normal colon tissues. (b)-(c) The occludin and Zo-1 expression levels decreased significantly in the stercoral obstruction group, compared with that of paired obstruction-adjacent normal colon tissues. (d)–(f) Serum levels of zonulin, IL-6, and TNF-*α* rose in the acute stercoral obstruction group, compared with volunteer.  ^*∗*^*P* < 0.05 independent experiments are performed for each test.

## Data Availability

The simulation experiment data used to support the findings of this study are available from the corresponding author upon request.
